This article has been retracted.

# Dual versus mono antiplatelet therapy for acute non- cardio embolic ischemic stroke or transient ischemic attack, an efficacy and safety analysis - updated meta-analysis

**DOI:** 10.1186/s12883-020-01808-y

**Published:** 2020-06-03

**Authors:** Christessa Emille Que Albay, Frederick Gavril D. Leyson, Federick C. Cheng

**Affiliations:** Cardinal Santos Medical Center, 10 Wilson St. Greenhills West, 1502 San Juan City, NCR Philippines

**Keywords:** Acute ischemic stroke, Non-cardioembolic stroke, Dual antiplatelet, Mono antiplatelet treatment, Aspirin, Cilostazol, Ticagrelor, Clopidogrel, Dipyridamole

## Abstract

**Background:**

New evidence on the efficacy and safety of dual antiplatelet therapy for secondary stroke prevention have been realized in the recent years. An updated meta analysis was done to determine the effect of the various dual antiplatelets vs aspirin alone on recurrence rate of ischemic stroke, cardiovascular morbidity and mortality, and its safety profile as reported through major bleeding.

**Methods:**

PubMed, Cochrane and Science Direct data bases were utilized, RCTs evaluating dual antiplatelet vs mono antiplatelet therapy for acute ischemic stroke or transient ischemic attack within < 72 h from ictus were searched up to July 2019. Risk ratio at 95% confidence intervals were calculated to evaluate stroke recurrence, cardiac events and mortality, and major bleeding.

**Results:**

Sixteen randomized controlled trials with a population of 28, 032 patients were pooled into a meta-analysis. Dual antiplatelet therapy was significantly superior over mono antiplatelet therapy in the reduction of stroke (RR 0.75, 95% CI:0.68–0.83, *p* value< 0.00001) and composite events namely cardiovascular morbidity and mortality (0.73 95% CI: 0.65–0.82, *p* value < 0.00001), while bleeding events were noted to be not significant (1.22 95% CI: 0.87–1.70, *p* value = 0.25).

**Conclusion:**

In acute non-cardioembolic ischemic strokes or those who have suffered a transient ischemic attack, dual antiplatelet therapy was associated with efficacy in stroke recurrence and composite cardiac events, with a non-significant risk of major bleeding.

## Background

Ischemic stroke is by far the most common type of stroke, accounting for approximately 80–90% of all strokes [1]. According to World Health Organization (WHO), cerebrovascular accidents (stroke) are the second leading cause of mortality and the third leading cause of morbidity. It is a condition in which a region of the brain is deprived of blood flow which results to hypoxia of brain cells leading to cell death, thereby resulting to focal neurologic deficits depending on the area of damage. Transient ischemic attack, on the other hand, presents similarly with ischemic strokes but do not leave evidence of damaged tissue. Transient impairment of blood flow occurs which reverses spontaneously without intervention.

Stroke is the leading cause of long disability. In addition to the initial damage, progression of focal deficits result to unfavorable outcomes. In the past decades, intensive therapeutic and interventional strategies have been investigated to reduce disability and recurrence of stroke. According to Aoki, et al. intravenous thrombolysis, endovascular therapy and aspirin have played key roles in reducing stroke recurrence [2]. Lifted from several prospective randomized controlled trials such as the CHANCE [3] and POINT [4] trials, the addition of clopidogrel to aspirin significantly decreased neurologic deterioration in patients with acute non cardioembolic ischemic strokes. Other dual anti-platelet therapies have also been showed to positively impact the management of ischemic strokes which have given rise to several systematic reviews and meta-analysis of these drugs. However, subsequent pilot studies with a small population size, involving antiplatelet drugs such as ticagrelor and cilostazol when combined with aspirin did not confirm whether clinical outcomes of patients with acute stroke would improve. Two recent randomized control trials were published on the use of Cilostazol with Aspirin, and Ticagrelor with Aspirin vs Aspirin alone, which were not included in the May 2018 meta-analysis by Yang Y, et al., on Dual vs Mono Antiplatelet Therapy for Acute Non-Cardioembolic Ischemic Stroke or Transient Ischemic Attack. These two additional randomized controlled trials provided data that was used to update the current management of secondary prevention of acute ischemic stroke. Hence, the aim of this study was to present an updated systematic review involving several antiplatelets, combined with aspirin as a dual therapy vs aspirin alone in its effect to: a. recurrence of stroke in patients who have suffered from acute stroke b. composite events such cardiovascular morbidity (i.e. acute coronary syndrome) and mortality c. safety as measured through major bleeding, among patients who have suffered from an acute non cardioembolic stroke.

Recurrent stroke may occur in 10 to 20% of patients within 3 months after the first stroke, therefore secondary prevention of stroke is very important. To reduce this burden, antiplatelet therapy is a key component of the management of non-cardioembolic ischemic stroke and transient ischemic attack [5]. The AHA/ASA recommended antiplatelet agents over oral anticoagulation to reduce the risk of recurrent stroke and other cardiovascular events (class I); and selection of an antiplatelet agent individualized on the basis of patient risk factor profiles, cost, tolerance, relative known efficacy of the agents, and other clinical characteristics (class I).

Aspirin, an irreversible inhibitor of cyclooxygenase and blocks the production of thromboxane A2, has been used in many trials and was found out to have favorable efficacy on the reduction of recurrence of ischemic stroke [6]. However, incidence of increased risk of bleeding as evidenced from previous studies suggested to use an alternative therapy.

Clopidogrel inhibits the binding of adenosine diphosphate to its platelet P2Y_12_ receptor and the subsequent adenosine diphosphate-mediated activation of the glycoprotein (GP) IIb/ IIIa complex [6]. It has been proven to reduce ischemic events as reported from previous clinical trials. However, dual combination anti platelet therapies was associated with increased risk of bleeding.

Cilostazol a phosphodiesterase 3 inhibitor, has three main mechanism of actions. It has an anti-platelet, vasodilatory and anti-inflammation effect [7]. A newer antiplatelet which has a comparable effect in reducing secondary ischemic stroke and when used as dual anti platelet therapy has similar risk for bleeding compared to Aspirin or Clopidogrel monotherapy [5].

Ticagrelor, a reversible P2Y_12_ receptor antagonist, does not require conversion from pro drug to active drug in the liver [8]. Occurrence of ischemic stroke was less compared to Aspirin, more efficacious in large artery disease and no major difference in bleeding episodes. However, in the said trials there were higher discontinuation of the drug because adverse effects such as dyspnea [6].

Dipyridamole is a platelet aggregation inhibitor. It inhibits the cAMP-phosphodiesterase, promotes adenosine inhibition of platelet function by blocking reuptake and subsequent degradation of adenosine and potentiation of prostacyclin (PGI_2_) an anti-aggregation. It is usually combined with aspirin and has been used in patients who have suffered from an ischemic stroke or transient ischemic attack. Several results showed its potential effect as an antiplatelet therapy for non-cardioembolic ischemic stroke or TIA and may be superior to aspirin [6]. However, side effects of headache and twice daily dosing have been noted.

Given that antiplatelet agents act through a range of mechanisms, including platelet inhibition of thromboxane A2 production, inhibition of cyclic adenosine 3′,5′-monophosphate production, and inhibition of P2Y12 receptors, a combination of agents can produce more effective stroke prevention than single agents [5]. Dual antiplatelet therapy may provide synergistic effect of inhibiting different platelet pathways for its activation.

Current guidelines for the management of acute ischemic stroke and TIA recommend antiplatelet therapy—typically providing strong recommendations for the use of a single agent, most commonly aspirin. Clear benefit of dual antiplatelet therapy on recurrent stroke without evidence of important adverse effects, is likely to provide clear guidance for patients with high risk TIA and minor ischemic stroke and for the clinicians responsible for their care [9].

### Objectives

The general objective of this study was to determine the effect of the various dual antiplatelets (including ticagrelor and cilostazol) vs aspirin alone on recurrence rate of ischemic stroke, composite events: cardiovascular morbidity – acute coronary syndrome, and mortality, and its safety profile as reported through major bleeding. In this study, all randomized trials used had an acute stroke or transient ischemic attack time frame of less than 72 h (< 3 days).

### Statement of the problem

This study sought to answer the question: Among patients with acute ischemic stroke or transient ischemic attack, is dual antiplatelet therapy (including novel anti-platelet medications) vs mono antiplatelet therapy effective in reducing stroke recurrence, cardiac composite events and major bleeding?

### Definition of terms

Composite events – defined as cardiovascular events: Acute Coronary Syndrome or Cardiac related death.

Dual Antiplatelet therapy – use of two concomitant antiplatelet medications with different mechanisms of action.

Ischemic Stroke – caused by blockage of an artery or in rare instances, a vein, leading to a condition in which a region of the brain is deprived of blood flow which results to hypoxia of brain cells leading to cell death [1].

Major Bleeding – as lifted from GUSTO: Severe life threatening – Intracranial hemorrhage or bleeding causing hemodynamic compromise requiring intervention [10].

Mono Therapy Antiplatelet – use of a single antiplatelet medication.

mRS – Modified Rankin Scale which measures degree of disability or dependence after a stroke [11].

NIHSS – NIH Stroke Scale, a tool used to objectively quantify the impairment caused by a stroke [12].

Non – cardio embolic stroke – caused by a blood clot that develops in the blood vessels inside the brain [1].

Cardio – embolic Stroke – caused by a blood clot or plaque debris due to LV dysfunction or cardiac arrhythmia [1].

## Methods

### Search strategy

Preferred Reporting Items for Systematic reviews and Meta-analyses (PRISMA) guidelines for this meta-analysis was used.

Update of the previous ‘Dual versus mono antiplatelet therapy for acute non-cardioembolic ischemic stroke or transient ischemic attack’ published in Stroke and Vascular Neurology in 2016 was done. A total of 16 eligible studies up to May 2019 were included in this meta-analysis.

A comprehensive and systematic search was used to retrieve relevant studies using the following electronic databases: PubMed, ScienceDirect, and COCHRANE Library. Key terms utilized were ‘antiplatelet therapy’, ‘aspirin or ASA’, ‘clopidogrel or Plavix’, ‘cilostazol or Pletaal’, ‘ticagrelor or Brilinta’, ‘dipyradamole’, ‘dual antiplatelet therapy’, ‘dual antiplatelet treatment’, ‘glycoprotein IIb/IIIa antagonists’, ‘acute stroke’, ‘stroke’, ‘transient ischemic attack’, ‘TIA’, ‘randomized controlled trial’. An expanded search was used using Booelan operators and MESH. Searches were restricted to trials on humans and reported in the English language, but no limit on date was applied. Incomplete or missing data from studies was requested from the respective investigators or authors by e-mail.

The citations identified by the search strategy were evaluated for eligibility and was further reviewed for accuracy using the inclusion and exclusion criteria outlined in Table 1.

**Table 1:** Inclusion and Exclusion Criteria

Inclusion	Exclusion
• Published randomized controlled trial • Dual vs mono (aspirin) therapy antiplatelet using in adults ages > 18 with non-cardioembolic ischemic stroke or transient ischemic attack which presented within 48 h of symptom onset • Administration of medication/s within 72 h of the acute ischemic event • NIHSS scores < 22, and a premorbid modified Rankin Scale of 0–2 • Studies with at least one clinical end point assessed (i.e. stroke recurrence, cardiovascular events, bleeding risk) ◦ Cardiovascular events include MI and death from cardiovascular causes ◦ Bleeding risk was defined by the Global Utilization of streptokinase and tissue plasminogen activator for occluded coronary artery definition [10].	• Studies with cardioembolic stroke with a high-risk source as defined by TOAST criteria [13] • Studies with the population already under medication with anti-platelet agents or any anticoagulants before stroke onset • Studies with co-intervention of thrombectomy, population with pregnant patients, in congestive heart failure, with GI ulcers or malignancy within the past 5 years • Studies judged inappropriate for the study by the investigator (due to lack of access to data) • Studies where the mono therapy antiplatelet was other than aspirin.

The primary outcome of interest in this study involved the recurrence of stroke in patients who received antiplatelet treatment within < 72 h from onset of an acute non-cardio embolic stroke, determining the dual antiplatelet protective effect in the prevention of further disability.

Secondary outcome in this study were as follows:

- Outcome of cardiovascular morbidity (Acute coronary syndrome) and mortality using dual antiplatelet vs mono therapy with aspirin,
- The safety profile of dual therapy antiplatelet vs mono therapy with Aspirin as reported through major bleeding.

### Data extraction and quality assessment

For studies from Jan 2016 to June 2019, study quality as to 1) study design, 2) study characteristics which included the population, intervention, control, outcome, methodology and duration of study and 3) inclusion and exclusion criteria were independently assessed. Also, trials published in the subgroup data from 14 studies were used directly from the previous meta-analysis.

The following items were assessed [1]: random sequence generation [2]; allocation concealment [3]; publication characteristics [4], countries included in the study [5], enrolled population [6], blinding of participants, investigators and outcome assessors [7]; sample size randomized within 72 h of ictus [8], treatment duration [9], intention to treat analysis [10], completeness of follow up where a < 20% loss to follow up rate led to less bias [11], efficacy and safety outcomes [12], incomplete outcome data [13]; selective outcome reporting; and [14] any other bias (e.g. insufficient rationale, study design).

### Data analysis

Primary analyses were performed for each outcome, with trials subdivided by the different medications assessed. Relative risk and 95% confidence interval were calculated using the random effects model since interventions, event rates and trial designs were expected to fluctuate.

Between study and between subgroup heterogeneities were evaluated by calculating I^2^ statistic and Cochrane Q (X^2^) statistic. Funnel plots were performed to check for publication bias due to different sample sizes. Two-sided probability values < 0.05 were considered statistically significant. All data were analyzed using Cochrane Review Manager (REVMAN 5.3).

## Results

### Study selection

Fourteen of the sixteen studies in the previous meta-analysis were included. Those excluded were trials where in the monotherapy treatment was not aspirin for uniformity of the control drug. For updated relevant studies from Jan 2016 to June 2019, data base searching and citation tracking of references identified 53,082, by using boolean function and the search terms mentioned above, the search was then narrowed down to 50 studies. By reviewing title and abstract, 44 trials were excluded, and 6 randomized control trials were reviewed by full text for details, and 4 of which were excluded due to missing data wherein all channels to retrieve it were exhausted. Therefore, 2 eligible randomised controlled trial were identified. Both of which compared its efficacy and safety versus aspirin in patients with acute non-cardioembolic ischemic stroke or transient ischemic attack (Fig. 1).

**Fig. 1:** Study Search Diagram based on the PRISMA Guideline

### Study characteristics

In total, there were 16 studies with 28,032 patients in the present meta-analysis (Additional file 1). Among which 12 were blinded studies, of which 9 were double blinded studies, 11 intention to treat and 15 had concealed allocation. Twelve trials enrolled patients with both ischemic stroke and transient ischemic attack while the remaining 4 trials enrolled patients with acute ischemic stroke. Onset to treatment intervals were < 24 h in 7 trials, < 48 h in 3 trials and < 72 h in 6 trials. The following antiplatelet medications were assessed in the meta-analysis: clopidogrel + aspirin vs aspirin (nine trials with 12,404 patients), dipyridamole + aspirin vs aspirin (five trials with 1037 patients), cilostazol + aspirin vs aspirin (two trials with 1284 patients) and ticagrelor + aspirin vs aspirin (1 trial with 13,307 patients).

### Quality assessment

Figure 2 presented the summary of the risk bias assessment of the studies used. Blinding evaluation was satisfactory in 14 of the 16 studies used, the remaining 2 studies were open labelled. Low risk bias was assigned to satisfactory blinded studies while high risk bias was assigned to open labelled studies.

**Fig. 2:** Summary of the risk bias assessment of the studies

Publication bias was analyzed using the funnel plots (Additional file 2). The study showed no significant publication bias by visual inspection of asymmetry in both the effect on recurrence of stroke and risk of bleeding, however scatter was not as significant in the composite events (Cardiovascular events and mortality plot).

Analyses of efficacy and safety outcomes showed that no evidence existed for between study heterogeneities with I^2^ values ranging from 6% (risk of recurrence of stroke), 18% (composite events: Cardiovascular events and mortality) and 22% (risk of bleeding). However moderate heterogeneities were seen between subgroups with I^2^ values ranging from 57.7% (risk of recurrence of stroke), 65.6% (composite events: Cardiovascular events and mortality) and 49.4% (risk of bleeding).

### Synthesis of results

Figure 3 presented the data regarding the efficacy outcome of stroke recurrence. Sixteen studies were analyzed, each of which have varying follow up durations, with insignificant attrition rates of < 10%, these studies were consistent in showing that dual antiplatelet significantly reduced the recurrence of stroke in patients who have suffered an acute stroke event or transient ischemic attack by 25% as compared to monotherapy (RR 0.75, 95% CI:0.68–0.83 at *p* value< 0.00001). Among the subgroups for dual anti-platelet, a comparable risk reduction was seen with using Clopidogrel plus Aspirin vs Aspirin yielding 33% significant reduction (9 studies: 0.67 95% CI: 0.58–0.76, *p* value< 0.00001), Dipyridamole plus Aspirin vs Aspirin with a 39% risk reduction (3 studies, 0.61 95% CI: 0.34–1.11, *p* value = 0.11) and Cilostazol plus Aspirin vs Aspirin showing a 34% risk reduction (2 studies, 0.66 95% CI: 0.27–1.63, *p* value = 0.37) in the recurrence of stroke. Although less reduction was seen in the Ticagrelor plus Aspirin vs Aspirin subgroup, a 14% significant reduction (1 study, 0.86 95% CI 0.75–0.99, *p* value = 0.04) was still evident.

**Fig. 3:** Forrest Plot on Efficacy Outcome of Stroke Recurrence

In Fig. 4, the use of dual antiplatelet over mono antiplatelet therapy showed a significant reduction in composite events such as cardiovascular events, acute coronary syndrome and cardiac associated deaths by 27% (0.73 95% CI: 0.65–0.82, *p* value < 0.00001) as generated from 11 studies. Subgroup analysis showed that 7 studies using Clopidogrel plus Aspirin vs Aspirin had a significant reduction of 31% in composite events (0.69 95% CI: 0.6–0.78, *p* value < 0.00001) and 2 studies presented the significant benefit of Dipyridamole plus Aspirin over Aspirin alone by 36%, (0.64 95% CI 0.38–1.08, *p* value =0.09). No significant risk reduction was seen in the Cilostazol plus Aspirin vs Aspirin Arm (1.0 95% CI: 0.45–2.25, *p* value = 1) while the use with ticagrelor over aspirin alone showed a harmful effect of increased composite events by 18% (1.18 95% CI: 0.83–1.69, *p* value = 0.35).

**Fig. 4:** Forrest Plot on Reduction in Composite Events (Cardiac related mortality and ACS)

Lastly, from the 14 studies utilized in examining the risk of bleeding and safety profile of dual antiplatelet therapy over mono antiplatelet therapy as presented in Fig. 5, increased major bleeding events were evident in dual antiplatelet therapy group by 22% (1.22 95% CI: 0.87–1.70, *p* value = 0.25). Subgroup analysis showed a 100% increase in bleeding risk with the use of Clopidogrel + Aspirin vs Aspirin alone (9 studies, 2.0 95% CI: 1.16–3.45, *p* value = 0.01) and a 29% increased risk of major bleeding in the Cilostazol + Aspirin regimen vs Aspirin alone (1.29 95% CI: 0.32–5.25, *p* value 0.33). Dual antiplatelet therapy using Dipyridamole + Aspirin vs Aspirin alone conferred an 8% reduced risk in major bleeding (2 studies, 0.92 95% CI: 0.06–14.76, *p* value 0.95) while the use with Ticagrelor over Aspirin alone had an 18% reduced risk in major bleeding (1 study, 0.82 95% CI: 0.51–1.32, *p* value = 0.41). Although increased risk of bleeding has been shown in the use of dual antiplatelet therapy, these values were not statistically significant since all *p* values were more than 0.05.

**Fig. 5:** Forrest Plot on Safety: Major Bleeding

Table 2 presented the comparison of data from 2018 meta-analysis of Yang, et al. and this current meta-analysis. Consistent evidence of significant decreased stroke recurrence and cardiac composite events (ACS and cardiac mortality) were seen with the use of dual antiplatelet therapy. Decreased stroke recurrence risk by 69% for Yang et, al. study and 75% for Albay, Leyson study were seen, while decreased cardiac composite events by 72% for Yang et, al. study and 73% for Albay, Leyson study were presented. There was a noted difference in major bleeding risk, a significant major bleeding risk was present in using dual antiplatelet therapy in the 2018 Yang Et, al study, which when studies with Cilostazol and Ticagrelor were added yielded a non-significant risk in major bleeding as presented in this meta-analysis.

**Table 2:** Comparison of Results from 2018 Dual vs Mono Antiplatelet Therapy and 2019 Meta-analyses

Results	Yang Et al. 2018 (RR; CI)	*P* value	Albay, Leyson 2019 (RR; CI)	*P* value
Stroke recurrence	RR 0.69, 95% CI: 0.61–0.78	< 0.001	RR 0.75, 95% CI:0.68–0.83	< 0.00001
Composite Events	RR 0.72, 95% CI: 0.64–0.80	< 0.001	0.73 95% CI: 0.65–0.82	< 0.00001
Major Bleeding	RR 1.77, 95% CI 1.09–2.87	0.02	1.22 95% CI: 0.87–1.70	0.25

## Discussion

Current guidelines for the management of acute ischemic stroke and TIA recommended antiplatelet therapy—typically providing strong recommendations for use of a single agent, most commonly aspirin [15–18]. The 2018 American Heart Association/ASA guidelines for management of acute ischemic stroke, stated a IIa recommendation on dual antiplatelet therapy on acute minor stroke [19, 20]. Given that antiplatelet agents act through a range of mechanisms – a combination of agents can produce more effective stroke prevention than single agents [21–24]. Dual antiplatelet therapy may provide synergistic effect of inhibiting different platelet pathways for its activation [25–28].

This research included recent studies on newer drugs like Cilostazol and Ticagrelor combined with Aspirin in preventing recurrent stroke, risk of cardiovascular events, mortality and risk of bleeding. These drugs showed promising results when combined with Aspirin in terms of their efficacy and prevention of composite events.

Studies have shown that Ticagrelor is independent of the genotypes that might affect antiplatelets activity, it was more efficacious than Aspirin or Clopidogrel whose efficacy were dependent on genetically determined metabolic activities. Cilostazol, on the other hand, has anti-platelet activity and multiple mechanisms of actions with vasodilatory, anti-inflammatory and anti-proliferative effects, because of which it has been recommended in other studies to be part of the standard of treatment [29]. Hence, with these newer drugs combined with the standard treatment of Aspirin, superior benefit in the management of acute ischemic stroke was achieved.

The use of Clopidogrel in previous studies has been proven to be more superior than Aspirin. This was in part due to the single pathway inhibited by Aspirin, thromboxane A2, which in turn, has little activity on Aspirin. While Clopidogrel inhibits two pathways – binding of adenosine diphosphate to its platelet receptor and the subsequent adenosine diphosphate mediated activity with glycoprotein complex (IIb/IIIa). Thus, when these two medications were combined, its synergistic effect potentiated prevention of a vascular event [16–18, 20, 23, 30]. However, the risk of bleeding episodes were statistically high with the dual antiplatelet therapy, although not statistically significant, when compared to mono antiplatelet therapy.

Studies and clinical trials on the use of Dipyridamole plus Aspirin has been established. Its efficacy and safety has not been superior compared to other drugs [22, 25, 27]. Hence, the investigators support the previous data of Dipyridamole plus Aspirin not being recommended as a standard of treatment due to its lesser efficacy and with no significant difference on bleeding risk.

The investigators were not able to further assess the other adverse effects aside from bleeding due to the limited studies employed from recent clinical trials and those with the newer developed drugs. Some adverse effects included difficulty of breathing associated with Ticagrelor; and palpitations or headache with Cilostazol use. However no noted life threatening adverse outcomes to date have been recorded.

There were certain limitations of this study that may have affected the interpretation of the results. First, duration of treatment and dosages varied among included studies though was rectified through assessing the heterogeneity via the I^2^ statistic. Second, evidence of some comparisons in terms of efficacy and safety with newer drugs were still limited and fewer smaller trials were conducted. Third, given the numerous subtypes of non cardioembolic ischemic stroke, efficacy analysis per subtype was not included in this study since most of the studies did not specify the subtype of non cardioembolic ischemic stroke, but only the severity of stroke. Hence, we recommend that further trials and studies be made on newer antiplatelets to establish their efficacy and safety, so that treatment guidelines can be established with lesser adverse events for the patient.

## Summary

Findings in this meta-analysis, can be summarized as follows: dual anti platelet therapy of any combination drug with Aspirin was statistically significant in reducing the recurrence of stroke, cardiovascular, and mortality events; safety in terms of any bleeding episode was not significant in using a dual antiplatelet or aspirin alone; among the dual anti-platelet therapy Clopidogrel plus Aspirin was the optimum dual therapy based on odds ratio for prevention of recurrent stroke, and cardiovascular events and mortality, but Clopidogrel plus Aspirin had the highest risk of bleeding episodes. Ticagrelor plus Aspirin was shown to be a promising drug combination in reduction of recurrence of stroke and composite events but its drawback was on its safety profile in terms of major bleeding events. Cilostazol with Aspirin can be a potential for optimal standard treatment due to its evidence in reduction of stroke recurrence, but with inadequate benefit as to composite events and increased risk of bleeding. By contrast, Dipyridamole plus Aspirin tend to be at par in efficacy in reduction of stroke recurrence with Cilostazol and Clopidogrel, but performed fairly in safety. As to cost, the most cost efficient combination was Cilostazol + ASA amounting to P29.5 pesos per day, followed Clopidgrel + ASA amounting to 39.5 pesos per day, then Ticagrelor + ASA amounting to 164.9 pesos per day [15]. (Additional file 3).

## Conclusion

Among patients with acute non-cardioembolic ischemic stroke or transient ischemic attack within 72 h of ictus, dual antiplatelet therapy was associated with a reduction in stroke recurrence and composite events such as Acute Coronary Syndrome and Cardiac related deaths when compared to monotherapy. However, dual antiplatelet therapy show a decreased safety profile due to the possible, although not statistically significant, events of major bleeding as observed in this study, factors that may have contributed to the increased risk of major bleeding were the dosing and duration of treatment given. In conclusion, the current data suggests that administration of short term dual antiplatelet therapy in the acute phase of ischemic stroke or transient ischemic attack was efficacious and relatively safe, of which Cilostazol with Aspirin can be a potential for standard treatment due to its evidence in reduction of stroke recurrence and being the most cost efficient combination although with not statistically significant bleeding risk.

## Recommendations

1. Further larger scale of clinical trials should be made on newer drugs (Ticagrelor and Cilostazol) to have a comparative power on efficacy over the optimal therapy and to address the safety or bleeding associated with Clopidogrel plus Aspirin.
2. Further studies on side effects on each anti platelet therapy should be made.

## Supplementary information

**Additional file 1.**

**Additional file 2.**

**Additional file 3.**

## Data Availability

All data generated or analysed during this study are included in this published article and its supplementary information files presented in the Appendices.

## Abbreviations

ACS: Acute Coronary Syndrome
ASA: Aspirin
AHA/ASA: American Heart Association / American Stroke Association
CHANCE: Clopidogrel in High Risk Patients with Acute Nondisabling Cerebrovascular Events trial
CI: Confidence Interval
GUSTO: Global Utilization of Streptokinase and Tissue Plasminogen Activator for Occluded Coronary Arteries
mRS: Modified Rankin Scale
NIHSS: National Institute of Health Stroke Scale
POINT: Platelet Oriented Inhibition in New TIA and minor ischemic stroke trial
PRISMA: Preferred Reporting Items for Systematic Reviews and Meta - Analyses
REVMAN: Review Manager 5
RR: Relative Risk
TIA: Transient Ischemic Attack
WHO: World Health Organization
